RETRACTED

# Molecular Phylogeny and Identification of the Peach Fruit Fly, *Bactrocera zonata,* Established in Egypt

**DOI:** 10.1673/031.011.17701

**Published:** 2011-12-31

**Authors:** Emtithal M. Abd-El-Samie, Zaki A. El Fiky

**Affiliations:** ^1^ Entomology Department, Faculty of Science, Cairo University, Giza 12613, Egypt; ^2^ Genetics Department, Faculty of Agriculture, Fayoum University, Fayoum 63514, Egypt

**Keywords:** mitochondrial cytochrome oxidase 1 gene (COI), restriction map, RT-PCR

## Abstract

The genetic structure of the Egyptian peach fruit fly (*Bactrocera zonata* (Saunders) (Diptera: Tephritidae)) population was analyzed using total RNA from adult females. A portion of mitochondrial cytochrome oxidase I (COI), 369 bp was amplified using RT-PCR, and was sequenced and analyzed to clarify the phylogenetic relationship of *B. zonata* established in Egypt. The data suggested that the gene shared a similarity in sequence compared to *Bactrocera* COI gene found in GenBank. Molecular phylogenetic analyses were performed based on nucleotide sequences in order to examine the position of the Egyptian population among many other species of fruit flies. The results indicate that four accession numbers of *B. zonata* (three from New Zealand and one from India) are closely related, while the Egyptian *B. zonata* are close to the 71 accession numbers of *Bactrocera* include one *B. zonata* from New Zealand. These two *B. zonata* from Egypt and New Zealand showed a close relationship in neighbor—joining analysis using the seven accession numbers of *B. zonata.* In addition, a theoretical restriction map of the homology portion of the COI gene was constructed using 212 restriction enzymes obtained from the restriction enzyme database to identify the Egyptian and New Zealand *B. zonata.*

## Introduction

Tephritid fruit flies in the genus *Bactrocera* (Diptera: Tephritidae) are distributed worldwide. The genus *Bactrocera* is a group of fruit flies containing more than 450 species (Drew and Hancock 2000; White 2000), and several *Bactrocera* species are serious pests of fruits and vegetables (Allwood et al. 1999). At least 28 *Bactrocera* subgenera have been denoted, and these are divided into four groups: *Bactrocera,* Melanodacus, *Queenslandacus,* and *Zeugodacus* (Drew 1989). The phylogenetic relationships among these *Bactrocera* species are poorly understood. Genetic markers and sequences from the mitochondrial genome in particular have proven informative in this respect (Shi et al. 2005; Xie et al. 2006). This is due to the availability of efficient PCR primers (Simon et al. 1994) and a wealth of comparative data (Jamnongluk et al. 2003b; Mun et al. 2003; Nardi et al. 2003; Reyes and Ochando 2004; Shi et al. 2005; Nardi et al. 2005; Boykin et al. 2006; Xie et al. 2006).

RETRACTED

Mitochondrial DNA (mtDNA) has been employed in phylogenetic relationships among tephritid fruit fly species, but the relationship among higher taxa could not be resolved (Han and McPheron 1997; Han 2000). Recently, by using 1.6 kb sequences of mtDNA, the more resolved phylogenetic relationship among higher taxa of the genus *Bactrocera* has been reported (Muraji and Nakahara 2001). The sequences of mtDNA contain the tRNA^leu^ and flanking cytochrome oxidase I and II (COI and COII) of regions (1.3 Kb) provide some useful perspectives on *Bactrocera* species relationships (Nakahara and Muraji 2008). Cytochrome oxidase I (COI) sequences were shown to be appropriate for intraspecific analysis because of the observed high degree of polymorphism. Furthermore, COI sequences have been used in some studies to address similar problems on a comparable geographic range, and using the same marker might facilitate comparisons (*B. depressa:* Mun et al. 2003; *B. dorsalis:* Shi et al. 2005; Nakahara and Muraji 2010; *Tetranychus urticae:* Xie et al. 2006). Additionally, PCR-RFLP-based methods of *Bactrocera* species identification was considered based on nucleotide sequences of the mtDNA (Muraji and Nakahara 2002). COI sequences are at the base of the barcoding identification system (Hebert et al. 2003); a valuable tool for species identification and discovery that has been proposed as a powerful methodology in biosecurity and invasive species identification (Armstrong and Ball 2005). A case study on tephritid fruit flies (Armstrong and Ball 2005) reported high rates of success, but also mentioned some difficulties with the identification of few species (e.g., *B. dorsalis, B. Cucurbitae, A. fraterculus*), where the occurrence of cryptic species, inadequate sampling of all genetic subgroups, and high levels of geographic differentiation might complicate identification.

The peach fruit fly, *B. zonata,* has been recognized as one of the most destructive flies attacking peach, apricot, guava, and figs (EPPO 2005). As this species is considered to be native to south and southeast Asia, it is thought to have been introduced to the Middle East, namely Saudi Arabia, Oman, and Egypt in recent years. Taher (1998) recorded this fly for the first time in Egypt, and it is now well— established, widespread, and well—adapted to local conditions (Hashem et al. 2001). Aedeagal length, body size, and number of pectin septa were used to distinguish between *B. zonata* found in Egypt with the sympatric species, *B. dorsalis* and *B. correcta* in Thailand (Iwahashi and Routhier 2001), and the study concluded that the aedeagal length can differentiate between these three species. A larger genetic distance was observed between populations of the peach fruit fly *B. zonata* collected from Thailand and Egypt than between many other pairs of distinctly different species (Nakahara and Muraji 2008). These populations were closely related with *B. correcta* in lineage clade (Muraji and Nakahara 2001; Nakahara and Muraji 2008), while *B. correcta* was close to *B. dorsalis* (Jamnongluk et al. 2003b). In this study, RT-PCR was performed to amplify a portion of the COI gene from *B. zonata* fruit flies established in Egypt. Comparative analysis of this sequence with *Bactrocera* COI genes found in the GenBank has been carried out to determine phylogenetic relationship. Moreover, a theoretical restriction map of COI fraction was performed to identify both the Egyptian and New Zealand *B. zonata* populations.

RETRACTED

## Materials and Methods

### Fruit fly collection and handling

The infested guava (*Psidium guajava* L.) fruits were collected from five locations (Abu Rawash, Badrashin, Ayyat, Imbaba, and El Saf) in Giza, Egypt during July 2008. Guavas were washed and placed in traps containing autoclaved sand. Fully—grown larvae of *B. zonata* that naturally jumped to the sand were allowed to pupate and rear to the adult stage in the laboratory at Cairo University, Giza, Egypt. Emerging adults were identified morphologically (E-*B.z.*) according to White and Hancock (1997). The identified female adults were rinsed in 70% ethanol, washed twice with double distilled water, dried using sterile tissue papers, and finally stored at -70 ^°^C for RNA extraction.

### RNA isolation and RT-PCR analysis

Total RNA was extracted from one female adult for each location using Gentra Purescript RNA Kit (www.qiagen.com). One µg of total RNA was reversely transcribed with RevertAid™ Minus Kit #K1631 (Thermo Fisher Scientific, www.thermoscientific.com) according to manufacturer instructions. PCR amplification was performed in 50 µL total volume with the following forward 5′ CATACGGATACAATGGTTAT 3′ and reverse 5′ TCGCGATCTGTCATATCCTG 3′ primers. PCR conditions were as follows: an initial denaturation step at 95 ^°^C for four min, 40 cycles of 94 ^°^C for 40 sec, 58 ^°^C for 40 sec, and 72 ^°^C for 40 sec, and a final extension step at 72 ^°^C for 10 min, using Perkin Elmer Gene Amp 9600 (www.perkinelmer.com). PCR products were checked by electrophoresis using 1.5% agarose gel in 1× TAE buffer. The products were then purified using QIAQuick Gel Extraction Kit #28706 (QIAGEN, www.quiagen.com) following manufacturer instructions and sequenced by automated DNA sequencing reactions, which were performed using a sequencing ready reaction kit (Life Technologies, www.invitrogen.com) in conjunction with ABI-PRISM and ABI-PRISM big dye terminator cycler.

RETRACTED

### DNA sequence and phylogenetic analyses

A consensus sequence of COI fragments from one female of each location was constructed by using the SeqMan™ II (Windows 32 SeqMan 4.05) package (DNAStar, www.dnastar.com). The sequence obtained in this study was submitted to the GenBank nucleotide sequence databases (Accession number: GQ225768). This sequence was subjected to alignment with COI sequences of the GenBank, EMBL, DDBJ, and PDB sequence database using the program BioEdit version 7.0.0 (Hall 1999). The PAUP version 4.Ob10 package (Swofford 2005) was used to generate a phylogenetic tree using the neighbor—joining methods based on Saitou and Nei (1987). A total of 500 bootstrap replicates were used for analysis.

### Identification of *B. zonata* established in Egypt

The restriction map of homology portion (57%) of COI of Egyptian *B. zonata* (accession number: GQ225768) was compared to three *B. zonata* (accession numbers: DQ116357, DQ116360, and DQ116361) (Armstrong and Ball 2005). The sequences were retrieved from NCBI as a GenBank file via their accession number by using NEBcutter program version 2.0 (Vincze et al. 2003). A restriction map was constructed using 212 restriction enzymes from a restriction enzyme database.

## Results

### Properties of DNA sequence

After amplifying cDNA, a single fragment of approximately 390 bp nucleotide sequences of the COI gene from five *B. zonata* female adults was amplified. Sequencing results exhibited that the total nucleotide length obtained from each one contained 390 bases. Alignments of these five sequences revealed 100% similarity between them. The DNA sequence compositions are 99 (A), 70 (C), 79 (G), 118 (T), and 3 (N). The nucleotide frequencies were 0.2538 (A), 0.3025 (T), 0.1794(C), and 0.2025 (G).

### Phylogenetic analysis

The topology of neighbor—joining tree and bootstrap support of the Egyptian *B. zonata* population (accession number: GQ225768) with 76 accession numbers of subgenus *Bactrocera* in the GenBank database represented a monophyletic group, bootstrap support < 50% (Figure 1). The three *B. zonata* fruit flies from New Zealand (accession numbers: DQ116357, DQ116360, DQ116361) and one from India (accession number: DQ838980) were clustered with each other showing bootstrap support < 50%, while *B. zonata* from New Zealand (accession number: DQ116359) was clustered with 72 fruit fly accession numbers of *Bactrocera* and showed bootstrap support 99%. The 72 accession numbers represented a monophyletic group with a 100% bootstrap support. Within this group, nine *B. umbrosa* fruit flies were closely related and formed a monophyletic lineage (100% bootstrap support). The Egyptian *B. zonata* population was found to cluster with 71 accession numbers of *Bactrocera* including *B. zonata* from New Zealand (accession number: DQ116358) (bootstrap support 100%); this accession number was found in a clade that consisted of *B. dorsalis* and *B. papayae* (bootstrap support < 50%).

RETRACTED

The seven accession numbers of the peach fruit fly *B. zonata* (Figure 1) were used to construct a phylogenetic tree of *B. zonata* (Figure 2). This tree represented a monophyletic group (bootstrap support < 50%) and the Egyptian *B. zonata* (accession number: GQ225768) showed a close relationship to *B. zonata* (accession number: DQ116358) from New Zealand (100% bootstrap support), while *B. zonata* (accession number: DQ116359) from New Zealand was closely related to the two previous accession numbers (90% bootstrap support). Two *B. zonata* fruit flies from New Zealand and India (accession numbers: DQ116357 and DQ838980, respectively) were closely related with each other (bootstrap support <50%) and to the three previous accession numbers (70% bootstrap support). The two *B. zonata* fruit flies from New Zealand (accession numbers: DQ116360 and DQ116361) were clustered with each other (bootstrap support < 50%).

### Identification of Egyptian *B. zonata*

A theoretical restriction map patterns of homology portion of COI using NEBcutter software program showed recognition sites of 22, 15, and 14 restriction enzymes in *B. zonata* from Egypt and New Zealand accesion numbers GQ225768, DQ116357, and DQ116360/ DQ116361, respectively (Figure 3). The map showed the presence of 32 cut sites in GQ225768 and 23 cut sites in DQ116357, DQ116360, or DQ116361. The DQ116357 differed in restriction enzymes SetI and Sth132I cut sites, whereas the DQ116360 and DQ116361 had the same restriction enzyme map. The restriction enzymes CstMI, HpyAV, Tsp509I, and TspDTI had the same restriction cut sites in the four accesion numbers, and the Egyptian *B. zonata* (GQ225768) differed in all other enzymes.

## Discussion

The adaptation to the environmental conditions produced by the host plants might play a role in speciation of tephritid fruit flies in the genus *Bactrocera* (Jamnongluk et al. 2003b). Total RNA of one *B. zonata* female for each location has been used to amplify a fragment of COI gene (390 bp). Alignment of these five sequences revealed 100% similarity between them. This similarity may be due to the fact that the five locations, which represent five districts at Giza governorate, have the same environmental conditions where the infested fruits were collected from the same host plant. Molecular analysis of the consensus sequence showed that the A+T content in Egyptian *B. zonata* population was 59%. These data are in agreement with the molecular analysis of Jamnongluk et al. (2003a) who reported that the A+T content of the 639 bp downstream segment of COI in species of the genus *Bactrocera* was slightly lower (63–68%) than those reported in other insects over the same segment; for example, 71% in *L. migratoria* (Flook et al. 1995), 69% in *An. gambiae* (Beard et al. 1993), and 70% in *C. capitata* (Spanos et al. 2000).

RETRACTED

The results clearly indicate that the four accession numbers of *B. zonata* (three from New Zealand and one from India) were closely related, while the Egyptian *B. zonata* (accession number: GQ225768) was close to the 71 accession numbers of *Bactrocera,* including other one *B. zonata* from New Zealand (accession number: DQ116358). The latter was found in a clade consisting of *B. dorsalis* and *B. papaya,* and the different *Bactrocera* species did not form a monophyletic lineage. This is in agreement with data obtained by Jamnongluk et al. (2003b), who reported that *B. correcta* was close to *B. dorsalis* when using COI. Muraji and Nakahara (2001, 2002) also reported the disagreement between morphological classification and molecular phylogeny.

In reality, many fruit fly species such as *B. dorsalis* and *B. carambolae* are very capable invaders; however, it is difficult to distinguish between them since they have overlapping host and geographic ranges with *B. verbascifoliae,* which is not a recognized pest. Some morphologically indistinct regulated species such as *B. philippinensis* and *B. papayae* have different host and geographic ranges. This is important information for assessing the specific risk and pathway involved. For example, with the fruit flies, COI could not confidently discriminate some of the species within the *B. dorsalis* complex, for which an additional gene region may be appropriate (Armstrong and Ball 2005). Phylogenetic analysis of COI sequences suggests that tephritid fruit fly species that attack cucurbit plants (*Asiadacus, Hemigymnodacus,* and *Zeugodacus*) were more closely related to each other than to fruit fly species of the subgenus *Bactrocera,* which attack plants of numerous families (Jamnongluk et al. 2003b). They also suggested that adaptation to the environmental conditions produced by the host plants might play a role in the speciation of tephritid fruit flies in the genus *Bactrocera.* Moreover, The Queensland fruit fly *B. tryoni* and a sibling species *B. neohumeralis* are sympatric and produce viable and fertile hybrids (Pike et al. 2003). These two species could not be clearly discriminated in both neighbor—joining and maximum parsimony analyses (Nakahara and Muraji 2008).

RETRACTED

When comparing these results with other studies addressing similar problems on phylogenetic relationships, it is possible to observe different levels and patterns of genetic differentiation. It is worth mentioning that the oriental fruit fly *B. dorsalis* showed higher variability in the COI sequences (5.94% of variable sites, compared to 1.15% in the melon fly) with almost no sharing of haplotypes among populations and only weak signs of differentiation in the westernmost samples (Shi et al. 2005). On the other hand, the pumpkin fly *B. depressa* shows equally high levels of genetic differentiation (4.14%) of variable sites, but with strong differentiation between Japanese and Korean populations (Mun et al. 2003). Host plant differences and geographic isolation could have played an important role in species differentiation within seven closely related species of *B. tau* complex (Baimai et al. 2000) and 52 sibling species of *B. dorsalis* species complex (Drew and Hancock 1994).

The phylogenetic analysis of the 77 accession numbers indicated that some species were placed within other species of *Bactrocera,* having weak bootstrap support even though the adults were morphologically distinct. Consequently, phylogenetic analysis of seven accession numbers of the peach fruit fly *B. zonata* from Figure 1 was used to indicate the relationship among these populations. This analysis showed a close relationship between *B. zonata* from Egypt and *B. zonata* (accession number: DQ116358) from New Zealand (100% bootstrap support). Moreover, the peach fruit fly *B. zonata* collected from Thailand and Egypt were closely related to *B. correcta* in the lineage clade by using rDNA (Muraji and Nakahara 2001; Nakahara and Muraji 2008).

Accuracy of identification is also dependent on reliability of the simple sequence similarity approach. In this case, a portion of the COI of Egyptian *B. zonata* poplation was selected, which is similar in sequence with the three *B. zonata* populations from New Zealand, to construct the theoretical restriction map. This map, produced by 28 restriction enzymes, was used to identify the peach fruit fly *B. zonata* from Egypt and New Zealand. As a result, recognition sites of several restriction enzymes have been found, which could be used in PCR-RFLP (i.e., restriction enzyme SetI). The PCR-RFLP analysis was used to identify *B. zonata* fruit flies (i.e., AseI was expected to differ among 16 of 18 species). The remaining two species, *B. dorsalis* and *B. philippinensis,* were expected to be discriminated by analyses using DpnI and MseI (Muraji and Nakahara 2002). Also, the restriction enzymes DraI and SspI have been used to recognize 44 haplotypes of *B. dorsalis* complex (Nakahara and Muraji 2010). In addition, this information could promote the development of a realistic system of *B. zonata* diagnostics based on PCR-RFLP analysis (useful for practical purposes such as field research) and quarantine inspection.

RETRACTED

## Conclusion

The sequence analysis of the isolated COI gene showed 100% similarity between the five sequences of *B. zonata* collected from five locations having the same environmental conditions and the same host plant. The properly rooted tree might indicate that most *B. zonata* samples form a single lineage of uncertain relationship (polytomy) with the Egyptian *B. zonata* and most other *Bactrocera* lineages. To resolve the disagreement between morphological classification and molecular phylogeny of fruit fly species in the future, we suggest that combined sequences from more than one gene (i.e., COI, non-transcribed region between COI and tRNA^leu^, cytochrome B, 16S rDNA, ITS1, and ITS2) could be used to identify the same species collected from the same host.

**Figure 1.** Neighbor—joining dendrogram of 77 fruit flies *Bactrocera* generated based on Saitou and Nei distances. Bootstrap confidence limits are shown adjacent the branches of clades supported in more than 50% of 500 replications. High quality figures are available online.

**Figure 2.** Neighbor—joining dendrogram of seven peach fruit flies *Bactrocera zonata* generated based on Saitou and Nei distances. Bootstrap confidence limits are shown adjacent the branches of clades supported in more than 50% of 500 replications. High quality figures are available online.

**Figure 3.** Homology portion theoretical restriction map of four *Bactrocera zonata* COI showing the recognition sites of 28 restriction enzymes. (A): DQ116360 (63–229bp) and DQ116361 (63–229bp), (B): DQ116357 (63–229bp) and (C): GQ 225768 (156–366bp). High quality figures are available online.

## **Abbreviations: **

PCR: polymerase chain reaction;
RT: reverse transcription;
RFLP: restriction fragment length polymorphism
UA
